The article "Research on Several Key Problems of Medical Image Segmentation and Virtual Surgery" was published in 2022. Journal: Contrast Media Mol Imaging.

# Research on Several Key Problems of Medical Image Segmentation and Virtual Surgery

**DOI:** 10.1155/2022/3463358

**Published:** 2022-04-11

**Authors:** Dan Luo, Yu Zhang, Jia Li

**Affiliations:** School of Mechanical Engineering, Shenyang University of Technology, Shenyang 110870, Liaoning, China

## Abstract

Medical images play an important role in modern medical diagnosis. Many clinicians make correct and appropriate diagnosis and treatment plans by means of medical images. With the development of science and technology, the application of medical image needs not only to simply read the image, but also to fuse advanced technology to analyze and process the image from a deeper level, such as the proposal of virtual surgery. Therefore, this article focuses on several key issues of medical image segmentation and virtual surgery. First, medical images are preprocessed by gray level transformation, interpolation, and noise elimination techniques. Second, level set model-based segmentation algorithm is adopted and improved. Finally, a constrained Delaunay tetrahedron method based on a point-by-point insertion method is proposed to reconstruct the tetrahedron mesh model. In order to eliminate the thin element, the tetrahedron mesh model is optimized. The simulation results show that this article improves the segmentation algorithm based on the level set model, which effectively improves the contradiction between the convergence accuracy and the convergence speed of the algorithm. The proposed tetrahedral mesh reconstruction algorithm realizes the generation of tetrahedral finite element meshes with complex boundaries and improves the quality of the volume model by optimizing the model.

## 1. Introduction

From the invention of X-ray in 1898 by Rontgen to the appearance of X-ray computed tomography in 1970s, the mode of medical diagnosis has changed greatly. Doctors' diagnosis relies more and more on visual image information. The emergence of magnetic resonance imaging (MR), positron emission computed tomography, and other imaging equipment has broadened the vision of doctors and brought great help to their diagnosis and treatment. Using computer graphics and image processing technology to extract and display three-dimensional image information can help medical staff simulate the treatment and operation process. The application of computer graphics and image technology to three-dimensional medical data mainly focuses on the visualization of three-dimensional medical images. The research of visualization and the rapid development of virtual reality technology have jointly promoted the development of virtual surgery technology [1, 2]. Virtual Reality (VR) technology combines multimedia technology with simulation technology to create a virtual environment with vivid audio-visual and tactile effects, which enable users to experience and interact in a natural way in the virtual environment to generate their own immersive feelings and experiences [3–5]. Therefore, in order to study how to design and construct an immersive virtual reality system, it is necessary to include computer graphics, image processing and pattern recognition, intelligent interface technology, artificial intelligence technology, multisensor technology, voice processing and audio technology, network technology, parallel processing technology, and high-performance computer system, etc. Virtual surgery system is the application of virtual reality technology in modern medicine. Zhu et al. proposed an algorithm based on image fusion to enhance the performance and robustness of image dehazing. Based on a set of gamma-corrected underexposed images, a pixel weight map is constructed by analyzing global and local exposures to guide the fusion process. The brightness spatial dependence of the fused image is reduced, and the color saturation is balanced during the dehazing process. The performance of the proposed solution is confirmed in both theoretical analysis and comparative experiments [6]. Combining the characteristics of CNNs and transformer, Li et al. proposes a dual encoder–decoder structure of X-shaped network (X-Net). It can be a good substitute for traditional pure convolutional medical image segmentation network. In the encoding stage, local and global features are simultaneously extracted by two encoders, convolutional downsampling, and transformer, and then fused by skip connections [7].

With the popularization and development of medical images in clinical diagnosis, the role of medical images goes far beyond the visual observation of their anatomical structures. It is necessary to accurately locate, segment, extract, and quantitatively analyze areas of interest such as anatomical structures and lesion areas with the help of computer and image graphics technology. It is further used in image registration, 3D reconstruction, surgical simulation, intraoperative navigation, radiation therapy planning, disease progression tracking, computer-assisted surgery, and other technologies. This undoubtedly has far-reaching significance for improving the utilization value of image data, and can greatly improve the accuracy and correctness of clinical diagnosis.

Image preprocessing is to separate each text image and hand it over to the recognition module for recognition. This process is called image preprocessing. In image analysis, the processing performed before feature extraction, segmentation, and matching are performed on an input image. Although there are hundreds or even thousands of image segmentation methods, owing to the complexity of human anatomy, there is irregularity of the shape of tissues and organs and the differences between individuals. The general image segmentation method directly applied to the medical image cannot obtain the ideal segmentation effect. Medical image segmentation is a difficult task, and there is still no general theory and method for medical image segmentation.

In the research and application of images, people are often only interested in some parts of the image, usually called the foreground, and the rest is usually called the background. Image segmentation is the technology and process of dividing the image into distinct regions and extracting the foreground. As an important part of medical image analysis, image segmentation plays an important role in a large number of medical image applications, such as tissue volume quantification, diagnosis, lesion location, anatomical structure research, treatment, partial volume correction of functional imaging data, and surgical operation combined with computer technology. The quality of image segmentation directly affects the final result of image analysis.

Three-dimensional reconstruction of medical images is to study how to construct three-dimensional geometric models of tissues or organs from two-dimensional sequence images acquired by various medical imaging devices and to render and display them on the computer screen “authentically.” These medical imaging techniques include computed tomography (CT), magnetic resonance imaging (MIR), ultrasound (US), positron emission tomography (PET), single photon emission tomography (SPECT), etc. Three-dimensional reconstruction of medical images can be used in surgical planning, simulation, plastic and prosthetic surgery, radiotherapy planning, anatomy teaching, and so on. At present, in the research of three-dimensional reconstruction of medical images, there are two main methods of geometric model construction: surface model and volume model. Surface model refers to the use of surface mesh model to represent the object of study. Volume model is constructed and represented by the corresponding two-dimensional unit filled with the whole model space.

With the development of science and technology, the application of medical image is needed not only to simply read the image but also to fuse advanced technology to analyze and process the image from a deeper level. Therefore, this article studies the segmentation technology in medical segmentation and virtual surgery and the three-dimensional reconstruction technology of medical image.

The innovations of this article are as follows: (1) Preprocessing medical images through grayscale transformation, interpolation, and noise removal. The principle of grayscale transformation is to stretch the grayscale values near the grayscale range and compress the grayscale levels far from the tissue according to the grayscale range of the tissue to be displayed. (2) The segmentation algorithm based on the level set model is adopted, and the algorithm is improved. The contradiction between the convergence accuracy and the convergence speed of the algorithm is effectively improved. (3) A constrained Delaunay tetrahedral mesh reconstruction method based on point-by-point interpolation is proposed. In order to eliminate thin elements, the tetrahedral mesh model is optimized, and the effective tetrahedral mesh model with complex boundaries is generated well, and the quality of the volume model is improved through optimization.

## 2. Proposed Method

### 2.1. Medical Image Preprocessing

#### 2.1.1. CT Value and Grayscale Transformation

Nowadays, CT machines are usually equipped with DICOM interface, which can be used to directly obtain the original data files of CT conforming to DICOM protocol. According to the imaging principle of CT machine, it is known that the CT value of the corresponding pixels is recorded in the data domain of data elements conforming to DICOM protocol, not the gray value of the general image.

CT value is a physical quantity indicating the attenuation degree of X-ray after passing through tissues. It is determined by the absorption coefficient *μ* of various tissues to X-ray. Based on the absorption coefficient *μ*_*H*_2_*O*_ of water, the formula for calculating CT value is shown in formula (1):

(1) $$\begin{array}{c} {\text{Value}}_{CT}=1000\times \frac{u_{X}-u_{H_{2}O}}{u_{H_{2}O}}. \end{array}$$

The principle of gray transformation in this article is to stretch the gray value near the gray range according to the gray range of the organization to be displayed and compress the gray level far away from it. Here, we introduce the concept of “window width” and “window position” in CT. If a CT value corresponds to the position of the gray-level center, then the CT value represents the window position. The window width indicates the range of CT values displayed.

Let *X* be the value of the original image pixels and *Y* be the value of the transformed image. The transformed *Y* value ranges from 0 to 255 gray scale, *L* is the center value of the window, and W is the width value of the window. The transformation formula is shown in formula (2):

(2) $$\begin{array}{c} Y=\left\{\begin{array}{cc} 0 & X\leq L-\frac{W}{2}\\ 255\; & X>L+\frac{W}{2}\\ \left(X-L+\frac{W}{2}\right)\times \frac{255}{W}, & L-\frac{W}{2}<X\leq L+\frac{W}{2} \end{array}\right.. \end{array}$$

Suppose the original image, consider each pixel, as an ant, then the ant includes the image's grayscale, gradient, and neighborhood features. The distance from any pixel is to expressed as Euclidean distance:

(3) $$\begin{array}{c} O_{ij}=\sqrt{\sum_{k=i}^{m}P_{k}{\left(X_{ik}-X_{jk}\right)}^{2}}. \end{array}$$

In formula (3), *m* is the dimension of the ant (*m* takes 3), and *p* is the weighting factor (which will be set according to the degree of influence of each component of the pixel). Let *b* be the clustering radius and be the pheromone, then we have

(4) $$\begin{array}{c} E_{ij}=\left\{\begin{array}{cc} 1, & E_{ij}\leq B\\ 0, & E_{ij}>B \end{array}.\right. \end{array}$$

At this time, if the path probability from to is selected as  *Pij*, then

(5) $$\begin{array}{c} P_{ij}=\left\{\begin{array}{cc} \frac{E_{ij}^{a}\left(t\right)n_{ij}^{b}\left(t\right)}{\sum_{s\in S}E_{is}^{a}\left(t\right)n_{is}^{b}\left(t\right)}, & j\in S\\ 0,\; & j\neq S \end{array}\right.. \end{array}$$

As the ants move, the pheromone on each path will change. After one cycle, the pheromone on each path is adjusted by the following formula:

(6) $$\begin{array}{c} E_{ij}\left(t\right)=\rho E_{ij}\left(t\right)+\Delta \rho E_{ij}. \end{array}$$

In the formula, *ρ* is the attenuation degree of the pheromone over time and is the increment of the path pheromone in this cycle:

(7) $$\begin{array}{c} \Delta \rho E_{ij}=\sum_{k=1}^{N}\Delta E_{ij}^{k}. \end{array}$$

In the formula, is the pheromone left in the path of the kth ant in this cycle. Let the selected initial cluster center be *Cj* (*V*; *G*; *Ne*), and the guiding function (the similarity between the pixel and the cluster center) is

(8) $$\begin{array}{c} n_{ij}=\frac{1}{d_{ij}}\\ =\frac{b}{\sqrt{\sum_{k=1}^{m}P_{k}{\left(X_{ik}-C_{jk}\right)}^{2}}}. \end{array}$$

The state of a single ant includes position information *r* and movement direction information *θ*. The transition probability of ants between different pixels is

(9) $$\begin{array}{c} W\left(\sigma \right)={\left(1+\frac{\sigma }{1+\delta \sigma }\right)}^{b}. \end{array}$$

Formula (9) is a two-parameter pheromone weighting function. The pheromone intensity of pixel *r* is *σ*(*r*), *β* is used to control the possibility of ants moving along the pheromone gradient direction, and 1/*δ* is the sensitivity of ants to pheromone. Taking into account, the inertia of the ant's motion, that is, the probability of its forward movement is relatively large. After adding a weighting coefficient  *W*(Δ*θ*), the transition probability of the ant from pixel *k* to *i* at time *t* is the following:

(10) $$\begin{array}{c} P_{ik}=\frac{W\left(\sigma_{i}\right)w\left(\Delta i\right)}{\sum_{j/k}W\left(\sigma_{i}\right)w\left(\Delta i\right)}. \end{array}$$

In formula (10), *j*/*k* is the neighboring pixel of pixel *k*. is the difference between the direction of pixel *i* relative to *k* at (*t*−1), and the previous movement direction of the ant. The pheromone release amount is the following:

(11) $$\begin{array}{c} T=n+p\Delta h. \end{array}$$

In formula (11), *n* is a constant release; *p* is a constant; when the same window is taken around pixels *k*, and *I* is the similarity of pixels between windows:

(12) $$\begin{array}{c} \Delta h=\;a\;\frac{\left|m_{1}-m_{2}\right|}{\max\left|m_{1}-m_{2}\right|}+b\frac{\left|\sigma_{1}-\sigma_{2}\right|}{\max\left|\sigma_{1}-\sigma_{2}\right|}+c\;\frac{S}{S\text{max}}\;. \end{array}$$

In the formula, (*a* + *b* + *c*) = 1. *m* is the average grayscale intensity of the window pixels. *σ* is the variance of the gray-scale intensity of the window pixels. *S* is the difference in the grayscale histogram of the window pixels:

(13) $$\begin{array}{c} A=\left\{x,U_{A}\left(x\right)|x\in X\right\}. \end{array}$$

A mapping *UA*: *X*⟶[0, 1] can be constructed, which is a membership function. In particular, a fuzzy relationship *ρ* defined on *X* is a subset of *X* × *X*, with

(14) $$\begin{array}{c} \rho =\left\{\left(x,y\right)\;U_{\rho }\left(x,y\right)|\left(x,y\right)\in X\times X\right\}. \end{array}$$

The fuzzy relationship *ρ* has reflexivity, symmetry, and transitivity and is an equivalent relationship. In image segmentation, the space *X* corresponds to the image pixel feature space, and the fuzzy subset A is the fuzzy classification relative to the segmentation target.

The basic idea of region growth is to merge pixels with similar characteristics into a certain region. First, determine a seed pixel as the starting point of growth for each region that needs to be segmented, as shown in Figure 1.

Then, according to certain growth criteria, the surrounding pixels with the same or similar characteristics are merged into the area where the seed pixels are located, and these new pixels are used as seeds to continue to grow as shown in Figure 2.

The segmentation process of the graph cut algorithm is shown in Figure 3. The solid line in the figure is n-links, and the dotted line is t-links. The source and sink points in the figure have been marked with S and T. The goal of graph cut is to find A secant line minimizes the addition of the cut t-link weight and n-link weight. After the segmentation is completed, it is divided into two parts, one part is only connected to the source point, and the other part is only connected to the sink point. The segmentation of the corresponding image is completed. In Figure 3(c), the green line is a secant, and 3(d) shows the final segmentation result.

The experiment template was established, and the traditional Hough transform detection algorithm and the straight line precision detection algorithm proposed in this chapter were used for comparative experiments. The detection results of the slope and intercept of the four straight lines are shown in Tables 1 and 2. After adding random noise on the four straight lines, Tables 3 and 4 show the corresponding test results.

In the absence of noise, the accuracy of the straight line detection algorithm proposed in this chapter is much higher than that of the Hough transform; after adding random noise, the accuracy of the improved algorithm decreases, but the accuracy is still higher than that of the Hough transform.

#### 2.1.2. Fault Interpolation

Tomographic images, such as CT and MRI, scan data are the intensity (gray) values of each slice position, and there is no data at the inter space of each slice. Sometimes, it is necessary to reconstruct the surface or three-dimensional structure of an object from some scanned slice data. Because of the insufficient number of slices, the third-dimensional information is lacking. The reconstructed image is often a very thin segment, resulting in severe distortion and loss of three-dimensional significance. At this point, we need to insert some layers into these layers. But the data of these new insertion layers are not directly from the actual test, but calculated by the algorithm with the existing layers. Sometimes an image wants to be observed from a particular angle or section. The observation plane may not pass through the original data lattice. At this time, gray interpolation is also needed for the display surface.

Three linear interpolation methods are commonly used in three-dimensional image interpolation, in which the nearest adjacent points are set as follows: *f*_000_, *f*_001_, *f*_010_, *f*_011_, *f*_100_, *f*_101_, *f*_110_, *f*_111_. Let *x*, *y,* and *z* denote the distance between the sampling point and the 000 point, then the value of the sampling point *f*_*pqr*_ is the following:

(15) $$\begin{array}{c} f\left(p,q,r\right)=\left(1-x\right)\times \left(1-y\right)\times \left(1-z\right)\times f_{000}+x\times \left(1-y\right)\times \left(1-z\right)\times f_{001}\\ +\left(1-x\right)\times y\times \left(1-z\right)\times f_{010}+x\times y\times \left(1-z\right)\times f_{011}\\ +\left(1-x\right)\times \left(1-y\right)\times z\times f_{100}+x\times \left(1-y\right)\times z\times f_{101}\\ +\left(1-x\right)\times y\times z\times f_{110}+x\times y\times z\times f_{111}. \end{array}$$

A total of seven linear interpolations are performed in three directions. The advantage of this algorithm is that it is fast, and the interpolation effect is better when the distance between adjacent two pieces is not large. Because its information is only related to the adjacent two sides, it is a local interpolation. In order to improve the accuracy, there are also points in 18 or even 26 domains for interpolation, which will cost more computing time and storage space, and the interpolation effect is only slightly improved. In general, the accuracy of cubic linear interpolation using points in eight domains is enough to meet the needs.

#### 2.1.3. Image Noise Cancellation

When the input image signal is mixed with noise, it is almost impossible to filter all the noise without losing the strength of the original signal. Therefore, there are two requirements for filtering: (1) to maximize signal loss, not to damage the contour and edge of the image and other important information; (2) to filter out as much noise as possible, so that the image is clear and visual effect is good.

Aiming at the particularity of sequential medical images, we have implemented two kinds of filters: one-dimensional spatial filtering and two-dimensional spatial filtering. Two-dimensional spatial filtering is for a single image, filtering on the two-dimensional *XY* plane of the image, and one-dimensional spatial filtering is for the sequence image, filtering in the one-dimensional *Z* direction of the sequence image. For sequential images, three-dimensional spatial filtering is theoretically feasible, but its time complexity and space complexity are very high. Therefore, the filtering operation in this article is divided into two steps. First, one-dimensional spatial filtering is carried out between sequential images, and then two-dimensional spatial filtering is carried out in a single image. In this way, on the one hand, the upper and lower correlation of sequence images is utilized, on the other hand, the high complexity of three-dimensional spatial filtering is avoided. Experiments show that this filtering method can achieve good results.

Two-dimensional spatial filtering is the central issue of filtering research. In this article, two-dimensional spatial filtering is discussed more, while one-dimensional spatial filtering principle is relatively simple. In one-dimensional spatial filtering, we use a median filter with a window length of 5. In the research of two-dimensional spatial filtering, this article adopts the commonly used neighborhood averaging method, which is a low-pass filtering method [8–10].

For each pixel in the image, take an area centered on it and replace the gray value of the pixel with the weighted average value of the gray level of each pixel in the area. This is the neighborhood averaging method. The specific method is to take a square area, called a smooth window or mask, which is a two-dimensional array of weights [11–13]. The filtering process is to slide the window on the image and update the gray value of the pixels facing the center of the window according to the following formula (4). When each pixel is scanned once, the smoothing of an image is completed. This is the simplest way to smooth the image on the real plane. Let *f*′(*i*, *j*) be an image to be smoothed. The size of the smoothing window is (*ZN* + 1) *x* (*ZN* + 1), and the value of *N* is usually 1 or 2. Then the smoothed image can be represented as follows:

(16) $$\begin{array}{c} g\left(i,j\right)=\frac{\sum_{u=-n}^{n}\sum_{v=-n}^{n}W_{uv}\cdot f\left(i+u,j+v\right)}{\sum_{u=-n}^{n}\sum_{v=-n}^{n}W_{uv}}, \end{array}$$

where *f*(*i*+*u*, *j*+*v*) represents the pixels corresponding to the smoothing window in the original image, *g*(*i* · *j*) represents the processed image, and *W*_*uv*_ is the weight value in the smoothing window. Sometimes, for convenience, the weight *W*_*uv*_ is normalized to make ∑_*u*=−*n*_^*n*^∑_*v*=−*n*_^*n*^*W*_*uv*_=1, so that formula (4) has only the remaining molecular terms. In addition, generally speaking, the bigger the window, the stronger the smoothing ability. However, the noise elimination degree and the attenuation degree of the original image signal are proportional to the size of the window, so it is not that the larger the window, the better. In practice, windows of 3 × 3 and 5 × 5 sizes are commonly used.

### 2.2. Medical Image Segmentation

This article studies segmentation and 3D reconstruction in medical image segmentation and virtual surgery. After grayscale transformation, interpolation and denoising preprocessing of the image, an improved level set model segmentation algorithm is used to achieve medical image segmentation. Image segmentation is to distinguish different meaningful regions in an image and determine their boundaries, so that the separated regions do not overlap and overlap, and there is only one belonging region for any point in the image. Image segmentation is mainly based on various features of the image, which mainly includes image gray, color, texture, local statistical features, spectral features, or some prior knowledge.

The medical image of the computer X-ray photography system is 12 Bit (4096 gray scale), the data volume of a CR is 8 MB, the data volume of an ultrasound image is 512 × 512 × 8 bit, and a digital X-ray photography system. The medical image data volume of the chest radiograph is 16 MB, and the data volume of a breast DR is 4096 × 4096 × 12 Bit.  Table 5 shows the data volume requirements for different medical images.

In clinical application, the imbalance of gray level has a great influence on image segmentation. If the adjustment of gray level before image segmentation will increase the complexity of processing tasks, it is not a good method. Now, we add the task of gray-level imbalance correction to the process of image segmentation, and the segmentation and gray-level correction are carried out simultaneously.

Local Binary Fitting (LBF) energy [14–16] model can well combine gray-level imbalance correction with segmentation algorithm, and improve the Piecewise Constant (PC) [17–19] model commonly used in segmentation. In the PC model, there are the following definitions. In the given image *I*: Ω⟶*R*^*n*^, Ω ⊂ *R*^*n*^ is the definition space of the image, and if C is a closed contour, then the local gray matching energy is the following:

(17) $$\begin{array}{c} E^{PC}\left(C,c_{1},c_{2}\right)=\lambda_{1}{\int_{\text{in}\left(C\right)}\left(I-c_{1}\right)}^{2}\text{d}x+\lambda_{2}{\int_{\text{out}\left(C\right)}\left(I-c_{2}\right)}^{2}\text{d}x+v\left|C\right|. \end{array}$$

Among them, *c*_1_ and *c*_2_ are the adjusted gray values of the partition area, which are the gray values of the interior of the contour, respectively, *λ*_1_ and *λ*_2_ are the weight parameters, respectively.

Considering that the gray value of a single pixel may deviate from its proper gray value due to noise or other factors, we need to take the pixels near the point into account to reduce the influence of this factor. Now, we introduce the energy function of the modified PC model with the Gauss kernel function *K*(*x*) to construct the energy of the LBF model. For a point *x* ∈ Ω in the image, the local energy is the following:

(18) $$\begin{array}{c} \varepsilon_{x}^{LBF}\left(C,f_{1}\left(x\right),f_{2}\left(x\right)\right)=\lambda_{1}\int_{\text{in}\left(C\right)}K\left(x-y\right){\left|I\left(y\right)-f_{1}\left(x\right)\right|}^{2}\text{d}y\\ +\lambda_{2}\int_{\text{out}\left(C\right)}K\left(x-y\right){\left|I\left(y\right)-f_{2}\left(x\right)\right|}^{2}\text{d}y. \end{array}$$

The Gauss kernel function *K*(*x*) is defined as follows:

(19) $$\begin{array}{c} K_{\sigma }=\frac{1}{{\left(2\pi \right)}^{1/2}\sigma }e^{-{\left|x\right|}^{2}/2\sigma^{2}}. \end{array}$$

Such a Gauss kernel function satisfies the following conditions:

(20) $$\begin{array}{c} \left(1\right)\;K\left(-x\right)=K\left(x\right),\\ \left(2\right)\text{ When }\left|x\right|>\left|y\right|K,\left(x\right)\leq K\left(y\right),\text{ and }\left|x\right|⟶\infty ,K\left(x\right)⟶0,\\ \left(3\right)\int_{-\infty }^{\infty }K\left(x\right)\text{d}x=1. \end{array}$$

Now, that the local energy of each point is obtained, the global energy is the following:

(21) $$\begin{array}{c} \varepsilon^{LBF}\left(C,f_{1},f_{2}\right)=\int_{\Omega }\varepsilon_{x}^{LBF}\left(C,f_{1}\left(x\right),f_{2}\left(x\right)\right)\text{d}x+v\left|C\right|. \end{array}$$

Now, we rewrite the energy function represented by the above formula into the level set form, so that we can judge the outline from the level set function, then the local energy of any point can be rewritten as follows:

(22) $$\begin{array}{c} \varepsilon_{x}^{LBF}\left(\phi ,f_{1}\left(x\right),f_{2}\left(x\right)\right)=\lambda_{1}\int K\left(x-y\right){\left|I\left(y\right)-f_{1}\left(x\right)\right|}^{2}H\left(\phi \left(y\right)\right)\text{d}y\\ +\lambda_{2}\int K\left(x-y\right){\left|I\left(y\right)-f_{2}\left(x\right)\right|}^{2}\left(1-H\left(\phi \left(y\right)\right)\right)\text{d}y. \end{array}$$

Then, for the global energy function, we rewrite it into the form of level set function and get it:

(23) $$\begin{array}{c} E\left(\phi ,f_{1},f_{2}\right)=\varepsilon^{LBF}\left(\phi ,f_{1},f_{2}\right)+\mu P\left(\phi \right)+vL\left(\phi \right)\phi , \end{array}$$

where *P*(*ϕ*)=∫_Ω_(1/2)(|∇*ϕ*| − 1)^2^d*x* 和 *L*(*ϕ*)=∫_Ω_*δ*(*ϕ*(*x*))|∇*ϕ*(*x*)|d*x*.

For most active contour models, how to locate the target contour quickly and accurately is the main improvement of the algorithm. But in the general algorithm, if we need to speed up the algorithm, we need to increase the time step, but in this way, the contour cannot converge to the target boundary, resulting in erroneous results. If we want to locate accurately, we need to reduce the time step, so the convergence speed will be reduced correspondingly, affecting the speed of the algorithm. Here we use the method of variable time step to reconcile this contradiction, as shown in formula (21).

(24) $$\begin{array}{c} \tau \left(x\right)=\tau_{0}g\left(x\right),\\ g\left(x\right)=\frac{1}{0.5+\left|\nabla K*I\left(x\right)\right|}+1, \end{array}$$

where *τ*(*x*) is the time step we used, *τ*_0_ is the time step commonly used in the level set algorithm mentioned above, *K* is the Gauss kernel function, so that the flatter region in the image *g* (*x*) is larger, so the time step will become larger, and in the position of the larger gradient *g* (*x*) is close to 1, so recovery becomes the common time step. Because of the large gradient at the edge of the image target, only when approaching the edge of the target can the time step become smaller to slow down the evolution speed to improve the evolution accuracy. At the distance from the edge of the target, the time step will become larger to improve the evolution speed. Therefore, with such a time step, time can be focused on determining the boundary, which can not only accelerate the evolution speed but also ensure the accuracy of the problem.

### 2.3. Three-Dimensional Reconstruction of Medical Images

#### 2.3.1. Generation of Delaunay Tetrahedron Mesh by Point-by-Point Insertion Method

The algorithm is an extension of the point-by-point insertion method proposed by Watson in three-dimensional space. The idea of the algorithm is to define an initial mesh containing all the nodes, insert a node into the mesh, and find out the tetrahedral elements containing all the outer spheres. These elements are deleted to form a cavity containing inserting nodes, which are connected with each triangular surface of the cavity to form a new tetrahedral mesh. Repeat this process until the end of the partition, and finally delete the invalid tetrahedron.

The steps of point-by-point insertion are as follows:

(1) The initial mesh can be used to construct a tetrahedron element with a large enough set of known points. An appropriate choice is to make the inner receptacle of the tetrahedron element an outer receptacle of a bounded box with axially aligned points. The reason for this is to ensure that the deletion of the relevant units containing the vertices of the outsourced large tetrahedron unit does not lead to the deletion of tetrahedrons that should not be deleted when inserting a known set of points.
(2) The outsourced tetrahedron is added to the tetrahedron mesh as the first subdivision tetrahedron.
(3) Insert other input points, insert one at a time, and process as follows:
  1. Search all tetrahedrons in the tetrahedron mesh and find those tetrahedrons whose outer spheres contain insertion points.
  2. Delete all the tetrahedrons in the previous step and form a cavity. Connect the inserted points with the boundary of the cavity to form a new tetrahedron element.
(4) When all points are inserted, the relevant tetrahedral elements containing the vertices of outsourced large tetrahedral elements are deleted, and the resulting meshes are the Delaunay tetrahedral subdivision of these points.

According to the characteristics of Delaunay triangulation, if the boundary of the three-dimensional data domain is convex, the data domain will be able to achieve Delaunay triangulation with the same boundary. Because of the complexity of human tissue, there are both convex and concave surfaces. The tetrahedral mesh generated by this algorithm has the problem of boundary inconsistency mentioned above. To solve this problem, we introduce a three-dimensional constrained Delaunay tetrahedral method to solve the problem of boundary inconsistency effectively.

In order to enable the PACS server to meet the requirements of image information flow at any time and ensure the data throughput capacity of the system, it is necessary to design the prefetching and preallocation scheduling control mechanism of the PACS, so as to avoid the overload and even paralysis of the network caused by the peak use of the system.  Figure 4 shows the distribution of the hospital's daily peaks of patient image information call.

#### 2.3.2. Three-Dimensional Constrained Delaunay Tetrahedron

The so-called “constrained Delaunay tetrahedral” subdivision refers to the tetrahedral subdivision based on Delaunay criterion under certain conditions. Constraints refer to the existence of boundary edges and boundary surfaces in a three-dimensional model. The following steps are given for the constrained Delaunay tetrahedral algorithm:

1. Read the boundary points, interior points, and the initial division of the boundary (obtained from the reconstructed surface model).
2. The constraints of partition are obtained from the initial partition of boundary, that is, the set of constrained edges and the set of constrained triangular surfaces.
3. Delaunay triangulation is performed for boundary points and interior points using the point-by-point insertion algorithm in the previous section.
4. Detecting which boundary edges and boundary surfaces are lost.
5. Restoration of constrained edges.
6. Restoration of constraint surface.
7. Using the dyeing method [20–23] to delete the useless units outside the entity and get the final segmentation results.

#### 2.3.3. Elimination of Silver Tetrahedron Thin Element

Canvendish divides Silver tetrahedral units into two categories in his article. The first one is that there are two common nodes in the four adjacent tetrahedrons of Silver element. Assuming that ABCD is a Silver element, its four adjacent tetrahedrons are ACDE, ABCE, BCDG, and ABCE, respectively. Among them, ACDE and ABCE have a common node E. For this kind of Silver element, elimination method is very simple, as long as the deletion method is adopted, the Silver tetrahedral element ABCD will be deleted from the tetrahedral grid, the original two elements ACDE, ABCE into BCDE, ABDE. In fact, after a local transformation, Silver tetrahedron elements are deleted without affecting the quality of all its adjacent tetrahedrons.

The second type is that there are no two common nodes in the four adjacent tetrahedrons of the element, and ABCD is a Silver element. There are no two common nodes in the four adjacent tetrahedrons of the element. At this time, the problem cannot be solved by deleting the Silver element directly. If the Silver element ABCD is deleted directly, the topological relationship between the remaining adjacent elements cannot be guaranteed, resulting in incompatibility of the generated grid topology. Canvendish's method is to move one of the four nodes A, B, C, and D, that is, to “pull” the flat unit ABCD. When pulling, it should be noted that the node cannot be pulled at will, otherwise, it may lead the mobile node to the interior of other cells and lead to the error of intersection of cells.

## 3. Experiments

In order to measure the performance of the filtering algorithm, the signal-to-noise ratio (SNR) [24, 25] is introduced to evaluate the filtering effect of the algorithm. The lower the signal-to-noise ratio, the worse the signal quality; the higher the signal-to-noise ratio, the better the signal quality [26]. One of the purposes of filtering is to improve the signal-to-noise ratio of signals. The formula for calculating SNR is as follows:

(25) $$\begin{array}{c} SNR=10\;\log\left(\frac{PS}{PN}\right). \end{array}$$

PS and PN represent the effective power of signal and noise, respectively.

In this article, human brain image is segmented by segmentation algorithm [27]. The simulation data used in the experiment are provided by McConell Brain Imaging Center and Montreal Neuroscience Research. The simulation data are generated by a MR simulator, which allows some imaging parameters (noise, offset field, etc.) to be independently adjusted. The advantage of this method is that it can test the algorithm quantitatively in different environments by using different quality images. The real segmentation of this model is expressed in the form of membership functions, which represent the probability that each voxel belongs to different classes. Only white matter, gray matter, and cerebrospinal fluid member functions were used in the experiment. In order to evaluate the experimental results, a criterion is needed to quantitatively represent the results. The Internet brain segmentation database provides an average coincidence measure to evaluate the segmentation results. Now let us briefly introduce: for any type *T*, *V*_*m*_ represents the set of artificially segmented voxels belonging to *T*, *V*_*α*_ represents the set of automatically segmented voxels belonging to *T*, then the average coincidence measure is defined as the ratio of the total number of voxels belonging to both segmentations, expressed in mathematical form as follows:

(26) $$\begin{array}{c} AOM=2\cdot \frac{\left|V_{m}\cap V_{\alpha }\right|}{\left|V_{m}\right|+\left|V_{\alpha }\right|}. \end{array}$$

The population size in SEA and DGEA algorithms is 100, while the population size in JSVH, SIHV, and ROSN are all 20. The dimension of particles in all algorithms is 30, and the maximum number of iterations is 2000. Each instance was run independently for 100 times, and the average optimal objective function value and variance were recorded in Table 6.

It can be seen from Table 7 that no matter which of *β* or *α* is equal to a fixed value, when the other is linearly reduced from 0.8 to 0.5, ROSN can have the best search accuracy. You can keep *β* between [0.8, 0.5] and decrease linearly, and let *α* be equal to a different fixed value and test again to finally determine the value of *α*. The test results are shown in Table 8.

In the experiment and simulation work of this article, the hardware configuration of the computer is as follows:

1. Processor: Inter i5 2.50 GHz
2. Memory: 4 GB
3. Operating system: Windows 7 64 ultimate
4. The simulation software is matlab 2016b

## 4. Discussion

Before medical image segmentation, image preprocessing is needed to enhance image quality. First, human brain CT images are transformed into gray images, which are shown in Figure 5(a). This is due to the wide range of CT values of medical image data, and image pixel data are generally stored in 16-bit integers. Gray-scale display devices are generally 8-bit, that is to say, image pixel data must be converted to 8-bit range before display. The image display mapped directly from 16 bits to 8 bits in the whole range will lose its diagnostic value. Therefore, a series of algorithms are needed to convert the original image data to the displayed image data.

Since the imaging principles of the endoscope and the camera are similar, in order to accurately and effectively calibrate the stereoscopic endoscope, the two-step calibration method of Zhang Zhengyou is used to separately calibrate the internal and external parameters of each camera. The multiple images of the calibration grid captured by the camera from different angles are collected and analyzed to solve the internal and external parameters of the camera. Endoscope calibration is the process of solving the spatial transformation matrix Treg of the stereoscopic endoscope video in Figure 6.

Then the gray image is equalized, and the processed image is shown in Figure 7(b). If the gray level distribution of the image is not uniform, the gray level distribution is concentrated in the narrow teaching range, which makes the details of the image not clear enough and the contrast is low. Therefore, image equalization can be used to make the gray scale of the image an open or an even distribution, so as to increase contrast, make the details of the image clear, and thus enhance the quality of the image. As can be seen from Figure 7(b), compared with the gray-level image in Figure 7(a), the image equalization process makes the image stretch nonlinearly and redistributes the gray value of the image, so that the gray level of the image in a certain range is approximately equal.

First, this article uses one-dimensional spatial filtering (median filter) and two-dimensional spatial filtering (domain averaging) to filter the image. The results are shown in Figure 5, where Figure 5(a) is an equalized image with noise and Figure 5(b) is a result image after filtering. It can be seen from Figure 5(a) that compared with Figure 7(b), the image information blurred by adding noise is disadvantageous to the subsequent image processing; from Figure 5(b), it can be seen that the image blurring is improved after filtering, and the image information is effectively restored to avoid the noise in the process of processing affecting the subsequent image segmentation.

In order to express the quality of the filtered image more clearly, the signal-to-noise ratio (SNR) is introduced as an evaluation index. The data of SNR before and after filtering are shown in Table 9. From the data in Table 9, we can see that after filtering, the signal-to-noise ratio of the image is increased by 11.35, which shows that the filtering process can effectively enhance the information of the image and provide better image quality for subsequent processing.

If the medical image processed by the improved ACO segmentation algorithm is lower than the quality of the random additional data of the imaging device, it is required to indicate whether the difference in quality will affect the clinical diagnosis. The readers use the naked eye to compare the quality of the medical image processed by the ACO segmentation algorithm and the quality of the random additional data of the imaging equipment, as shown in Table 10.

Table 11 shows the results of two image readers using the improved ACO segmentation method to evaluate the quality of 200 images and the quality of random additional data.

Table 12 shows the results of two film readers comparing the image quality of the 200-frame improved deformation model segmentation algorithm and the quality of random additional data.

There are 175 medical images with a score of “0,” that is, the quality of the two medical images is the same, accounting for 87.5% of all 200 medical images.

In this article, four groups of experiments were carried out from the simplest experiment, in which the voxel size was 1 mm. The noise of the first group of experiments is 3%, without migration field; the noise of the second group is 9%, which is used to test the robustness of the algorithm without migration field; the noise of the third group is 3%, and the migration field is 40%, which is used to test the robustness of the algorithm in the presence of migration field; the noise of the fourth group is 9%, and the migration field is 40%. The robustness of the algorithm in the case of noise and offset field. The experimental results are shown in Table 13. From Table 13, it can be seen that the AOM of white matter segmentation is stable at about 0.9, and that of gray matter segmentation is stable at about 0.79. Compared with the AOM of the first group and the second group, it can be seen that the robustness of the segmentation algorithm used in this article is very good when the noise is different. By comparing the AOM, of the first group and the third group, we can see that there is not much change to the AOM value after the migration field is added, and it is shown that the algorithm has good stability in the presence of the migration field. In addition, as long as *AOM* > 0.7, it is considered as a good segmentation, so the performance of the segmentation algorithm in this article is superior.

In order to better illustrate the advantages of this segmentation algorithm, this article uses the traditional K-means segmentation algorithm, FCM segmentation algorithm, KFCM segmentation algorithm as a comparison, comparing the data as shown in Table 14, drawing a broken line graph as shown in Figure 8.

Combining Table 14 and Figure 9, we can see that the lowest overall AOM value is K-means segmentation algorithm, which is 0.67, which is not a good segmentation algorithm; while FCM and KFCM are segmentation algorithms, the overall AOM values are 0.71 and 0.75, respectively, which can segment images well; the best overall AOM value is the proposed segmentation algorithm in this article, is 0.85, which shows the superiority of the segmentation algorithm in this article (Figure 10).

In order to verify the effectiveness of the fuzzy weighted entropy formula proposed in the article, this article selects medical images and ordinary images for comparison experiments. The comparison diagrams are shown in Figures 9, 11 and 12, and the respective normalized gray histograms are obtained as the graphs. 10, Figures 13 and 14.

The purpose of abdominal CT examination is to know whether there are infectious diseases in abdominal organs. As shown in Figure 9.

Compared with CT, brain magnetic resonance has the unique advantages of no radiation damage, no bone artifacts, multifaceted, and multiparameter imaging, high soft tissue resolution, and the ability to display vascular structures without the use of contrast agents. As shown in Figure 11.

The comparison results of liver CT are shown in Figure 15. It can be seen that the effect of this article is better and the picture is clearer.

The above three sets of experimental results show that the weighted entropy method proposed in the article is significantly better than the Cheng method and the Kapur method in various performances. At the same time, the weighted entropy method proposed in the article can also obtain better segmentation results for different types of images. Combined with the level set model segmentation algorithm proposed in this article, the parameter values are screened to select the appropriate parameter values.  Table 15 shows the parameters of the membership function and their cut-off values.

Image-based semantic segmentation is shown in Figure 16. The original image is a HE-stained pathological section of a mouse liver. Image segmentation is the process of dividing an image into several disjoint small local areas according to certain principles. It is one of the most basic research fields in image processing. At present, there are many image segmentation methods, among which the watershed algorithm is a region-based image segmentation algorithm. The watershed algorithm has been widely used in medical images, pattern recognition, and other fields because of its convenient implementation.

The c-means image segmentation with blurred local information is shown in Figure 17.

The image segmentation based on the watershed algorithm is shown in Figure 18. Watershed is a classical calculation method. The traditional watershed segmentation method is a mathematical morphological segmentation method based on topology theory. Representing the altitude of the point, each local minimum and its affected area is called a catchment basin, and the boundary of the catchment basin forms a watershed. The concept and formation of the watershed can be illustrated by simulating the immersion process.

## 5. Conclusion

Nowadays, it is very popular for doctors to make correct diagnosis by means of medical images, but simply staying at the level of reading images cannot meet the development of the times, more need to integrate advanced technology, more in-depth use of image processing technology, virtual surgery is a good way of application. In this article, the segmentation and three-dimensional reconstruction in medical image segmentation and virtual surgery are studied. After image preprocessing with gray-level change, interpolation, and noise elimination, the improved level set model segmentation algorithm is used to realize medical image segmentation. Experiments show that this method has good segmentation effect. By comparison with several traditional segmentation algorithms, the K-means segmentation algorithm has the lowest overall AOM value, which is 0.67, which is not a good segmentation algorithm. The overall AOM values of the FCM and KFCM segmentation algorithms are 0.71 and 0.75, respectively, which can segment the image well; the best overall AOM value is the segmentation algorithm proposed in this article, which is 0.85, which shows the superiority of the segmentation algorithm in this article. Then, a constrained Delaunay tetrahedron method based on point-by-point insertion method is proposed. On the basis of mesh reconstruction, the tetrahedron mesh model is optimized to eliminate thin elements effectively, and the tetrahedron effective element mesh model with complex boundary is well generated, and the quality of the volume model is improved by optimization. However, due to the limitations of experimental techniques, there are still some finer works that have not been studied in depth. For the automatic segmentation technology of medical images, we will continue to carry out further research and discussion.

## Figures and Tables

**Figure 1:** Setting the seed point.

**Figure 2:** Growth process.

**Figure 3:** The segmentation process of the graph cut algorithm.

**Figure 4:** Peak distribution of patient image information.

**Figure 5:** Filtering processing. (a) Image with noise. (b) Image after filtering.

**Figure 6:** Registration experiment scene and schematic diagram.

**Figure 7:** Gray level and equalization processing. (a) Grayscale image. (b) Image after equalization.

**Figure 8:** Performance comparison diagrams of several segmentation algorithms.

**Figure 9:** CT abdomen view.

**Figure 10:** CT abdomen histogram.

**Figure 11:** MRI brain map.

**Figure 12:** Lena diagram.

**Figure 13:** MRI brain map histogram.

**Figure 14:** Lena histogram.

**Figure 15:** The comparison results of liver CT(Some of the pictures are from Baidu).

**Figure 16:** Image-based semantic segmentation(Some of the pictures are from Baidu).

**Figure 17:** The c-means image segmentation with blurred local information (Some of the pictures are from Baidu).

**Figure 18:** The image segmentation based on the watershed algorithm(Some of the pictures are from Baidu).

**Table 1:** Comparison of straight line detection results without noise (slope).

Actual value		Traditional Hough		Improved detection method	
Line	Slope	Efficient	Relative error(%)	Efficient	Relative error(%)
A	0.63	0.65	3.60%	0.63	0.04%
B	0.23	0.25	11.19%	0.23	0.87%
C	0.72	0.74	3.25%	0.72	0.10%
D	−0.14	−0.11	23.45%	−0.14	0.78%

**Table 2:** Comparison of straight line detection results in noise-free condition (intercept).

Actual value		Traditional Hough		Improved detection method	
Line	Slope	Efficient	Relative error(%)	Efficient	Relative error(%)
A	0.33	0.37	10.69%	0.33	0.57%
B	0.36	0.39	8.74%	0.36	0.10%
C	−0.03	0.00	113.82%	−0.03	0.18%
D	−0.41	−0.37	9.02%	−0.41	0.03%

**Table 3:** Comparison of linear detection results with noise (slope).

Actual value		Traditional Hough		Improved detection method	
Line	Slope	Efficient	Relative error(%)	Efficient	Relative error(%)
A	0.11	0.14	26.57%	0.11	1.07%
B	0.39	0.41	5.31%	0.39	0.29%
C	0.58	0.62	6.40%	0.58	0.03%
D	0.69	0.72	3.99%	0.69	0.01%

**Table 4:** Comparison of linear detection results with noise (intercept).

Actual value		Traditional Hough		Improved detection method	
Line	Slope	Efficient	Relative error(%)	Efficient	Relative error(%)
A	0.53	0.56	6.97%	0.53	0.23%
B	0.61	0.64	4.99%	0.61	0.16%
C	−0.52	−0.50	5.22%	−0.52	0.21%
D	0.49	0.52	5.30%	0.50	0.29%

**Table 5:** Data volume of medical imaging image files.

Medical imaging image imaging type	Single image (bit)	Check the amount of file data required (MB)
Nuclear medicine	512 × 128 × 12 × (2)	57
MRI	256 × 1080 × 8 × (30)	31
Ultrasound	128 × 2048 × 12 × (2)	114
DSA	1080 × 512 × 8	53
X-CT	2048 × 256 × 12 × (2)	125
CR	4096 × 128 × 8 × (15)	44
DR	128 × 2048 × 8	45
Breast DR	2048 × 512 × 12	25

*Note.* The minimum number of images that can meet the diagnostic requirements is in parentheses.

**Table 6:** Average optimal objective function value and variance.

	SIHV	JSVH	ROSN	AIFN	DRQPSO	FS
Rosenbrock	459.53	673.22	491.59	533.97	533.67	480.11
(Std.Dev)	(158.96)	(184.18)	(651.92)	(215.04)	(507.72)	(317.30)
Rastrigrin	35.23	50.27	56.67	41.75	53.52	35.76
(Std.Dev)	(43.27)	(58.88)	(45.42)	(27.92)	(17.00)	(40.85)
Greiwank	0.31	0.17	0.31	0.18	0.21	0.62
(Std.Dev)	(0.57)	(0.34)	(0.41)	(0.26)	(0.59)	(0.23)

**Table 7:** Function test results when *α* linearly decreases and *β* = 0.6.

*α*	1⟶0.5	1⟶0.6	1⟶0.7	1⟶0.8	1⟶0.9
Rosenbrock	651.90	652.23	389.31	178.18	199.13
(Std.Dev)	(216.54)	(247.67)	(666.84)	(376.87)	(438.81)
Rastrigrin	45.79	47.65	36.04	21.90	48.85
(Std.Dev)	(67.41)	(50.46)	(26.23)	(50.90)	(27.95)
Greiwank	0.37	0.33	0.66	0.32	0.46
(Std.Dev)	(0.37)	(0.57)	(0.31)	(0.37)	(0.44)

**Table 8:** The function test results when *α* is equal to different fixed values and *β* decreases linearly within [0.8, 0.5].

*α*	0.2	0.3	0.4	0.5	0.6
Rosenbrock	548.54	229.00	422.18	473.16	395.82
(Std.Dev)	(314.51)	(577.48)	(400.12)	(176.68)	(647.22)
Rastrigrin	30.01	61.77	23.94	31.00	51.23
(Std.Dev)	(16.89)	(64.67)	(62.96)	(67.05)	(50.19)
Greiwank	0.32	0.28	0.36	0.53	0.55
(Std.Dev)	(0.58)	(0.23)	(0.38)	(0.56)	(0.31)

**Table 9:** Comparison of SNR data before and after filtering.

Image	SNR
Before filtering	8.77
After filtering	20.12

**Table 10:** Comparison of improved medical image segmentation algorithm quality and random additional data image quality.

	Physician A	Physician B	Statistics on the reading results of doctors A and B
Medical image a	+	+	++
Medical image b	+	0	+
Medical image c	+	—	0
Medical image d	0	+	+
Medical image e	0	—	—
Medical image f	—	0	--
…			
200 medical images			

**Table 11:** The improved ACO segmentation method image quality evaluation results statistics.

	Doctor A rated ++	Doctor A rated +	Doctor A rated 0	Doctor A rated -	Doctor A rated --
Doctor B rated ++	15	17	9	6	16
Doctor B rated +	16	3	2	9	4
Doctor B rated 0	3	4	15	10	6
Doctor B rated -	3	3	2	11	4
Doctor B rated --	12	13	9	5	3

**Table 12:** Image quality evaluation results statistics of improved deformation model segmentation method.

	Doctor A rated ++	Doctor A rated +	Doctor A rated 0	Doctor A rated -	Doctor A rated --
Doctor B rated ++	0	0	0	0	0
Doctor B rated +	0	8	175	0	0
Doctor B rated 0	0	1	12	1	0
Doctor B rated -	0	0	1	2	0
Doctor B rated --	0	0	0	0	0

**Table 13:** Segmentation of experimental AOM data.

Experimental grouping number	White matter	Gray matter	Whole
First group	0.92	0.77	0.85
Second group	0.93	0.81	0.87
Third group	0.89	0.79	0.84
Fourth group	0.87	0.80	0.84

**Table 14:** Performance comparison of several segmentation algorithms.

Segmentation algorithm	Whole AOM
K-mean segmentation algorithm	0.67
FCM segmentation algorithm	0.71
KFCM segmentation algorithm	0.75
Method in this article	0.85

**Table 15:** Membership function parameters and thresholds.

Picture	Method	a	b	c	T1	T2
CT map	Cheng method	47	41	39	57	26
	Kapur method	76	36	50	9	64
	Method of this article	10	83	10	31	64

MR chart	Cheng method	34	25	64	82	9
	Kapur method	13	85	30	87	9
	Method of this article	62	20	18	44	14

Lena diagram	Cheng method	43	75	78	73	5
	Kapur method	54	52	30	86	70
	Method of this article	49	8	49	46	42

## Data Availability

This article does not cover data research. No data were used to support this study.
